# Research on System Construction and Strategy of Intelligent Sports in the Implementation of National Fitness

This article has been retracted.

**DOI:** 10.1155/2022/3190801

**Published:** 2022-05-10

**Authors:** Yuxin Tang, Shengfeng Zan, Xiaowen Zhang

**Affiliations:** ^1^School of Physical Education, Shandong University, Jinan, Shandong 250061, China; ^2^School of International Studies, Renmin University of China, Beijing 100872, China

## Abstract

This paper studies the construction and development strategy of intelligent sports system in the context of Chinese National Fitness Program with methods of literature review and model construction. The research shows that there are four dilemmas in the implementation of intelligent sports in national fitness: data security, market monopoly, legal supervision, and product iteration. However, there are also three promoting factors in this regard, including policy guarantee, market demand, and industrial upgrading. Following the principles of scientificity, effectiveness, public welfare, and collaboration, this paper designs a system for intelligent sports in national fitness. The construction of the national fitness intelligent sports system mainly consists of four modules, including basic framework construction, function design, content design, and operation analysis. With the systematic analysis of the status quo of intelligent sports application in national fitness, this paper puts forward intelligent sports development strategies in the implementation of national fitness from four aspects: optimizing the top-level design of government, speeding up industrial transformation and upgrading, constructing market supervision mechanism, and establishing a talent training system.

## 1. Instruction

The “New Generation AI Development Plan” issued by Chinese State Council in 2017 marked that artificial intelligence(AI) would become a key national development field, and AI would be more applied to the real world, so as to improve the efficiency of industrial development, inject power into traditional industries, and promote new industrial reform. With the development of artificial intelligence in the field of sports in recent years, new breakthroughs have been made in sports intelligent manufacturing. As mentioned in the “Outline of Building a Sports Power” and “Opinions on promoting national fitness and sports consumption to promote high-quality development of sports industry,” China will accelerate the application of emerging technologies such as Internet Plus, big data, and artificial intelligence in the national strategy of national fitness, and promote the integrated development model of “sports plus.” It can be concluded from a number of national policies that the first step to develop national fitness in China is to encourage new forms of national fitness, improve sports consumption patterns, and upgrade the traditional industrial system. The second step is to promote the open sharing of national fitness data resources, improve the digital infrastructure and security guarantee of national fitness, and accelerate the innovative application of resources. Thirdly, it aims to focus on cultivating and strengthening digital sports economy, and promote digital transformation in all fields of national fitness. Finally, it aims to promote the in-depth implementation of the national strategy of fitness for all and open up a new prospect in building China into a sports power.

However, at present, intelligent sports is still in its infancy in the implementation of national fitness, and its application, integration, and development strategies still need further exploration and research. There are many problems in the development of intelligent sports in the national fitness: how to plan the infrastructure layout of intelligent sports in the national fitness? How to coordinate government departments, market, industry, and the public? How to better integrate intelligent sports into this national strategy? How to deepen the implementation of national fitness? It is particularly important to explore the development strategy of intelligent sports in the implementation of national fitness. Therefore, this article is going to construct an intelligent sports system in national fitness from both macro and micro perspectives, and conduct research on the content, function, and operation of this system. The analysis of the development path of intelligent sports can help intelligent sports better integrate and develop in the implementation of national fitness, achieve the best coupling of “sports + artificial intelligence,” and eventually promote the effective implementation of national fitness strategy.

## 2. Intelligent Sports: Rise, Development, and Application

### 2.1. The Rise of Intelligent Sports

Intelligent sports is a knowledge system which takes sports as the main body, and uses artificial intelligence, Internet, Internet of Things, big data, and other high-tech means to exert a certain influence on human body activities and sports thoughts. From a time perspective, intelligent sports and artificial intelligence emerged almost at the same time. In 1950, Alan Turing first proposed the concept of artificial intelligence based on the intelligence of machines [1]. In 1951, British scholar Christopher Strachey wrote a computer program about checkers, which opened the prelude to the rise of intelligent sports. In 1955, “A Proposal for the Dartmouth Summer Research Project on Artificial Intelligence” first proposed the concept of Artificial Intelligence, “to use computers to simulate human behavior and realize machine intelligence.” In 1956, the first special seminar on artificial intelligence was held in the United States. The successful application of knowledge engineering and expert systems in 1970–1980 laid the foundation for the development of artificial intelligence [2]. Deep Blue's victory over chess champion Garry Kasparov in 1997 marked a breakthrough for AI in sports. AI has experienced three waves including Turing Test, speech recognition, and deep learning [3]. With the continuous rise of intelligent sports, human beings have changed from physics-society (PS) to cyberspace-physics-society (CPS), forming a more complete ecosystem of artificial intelligence and human development, providing a theoretical basis for the rapid development of intelligent sports.

### 2.2. The Development of Intelligent Sports

The development of intelligent sports has become an important research field for scholars at home and abroad. Lapham and Bartlett [4] studied the performance prediction system of AI in sports events. AI's prediction of sports events can exceed human's prediction level [5]. Li and Zhang [6] conducted in-depth research on legal issues and development strategies in intelligent sports. Wang [7] analyzed the ethical dilemma caused by artificial intelligence on sports, and explained and interpreted it from a philosophical perspective. Yu and Gao [8] put forward the characteristics of automaticity, intelligence, and controllability for AI-assisted training, which is of great value in sports simulation training, sports detection, and other practices. In the 21st century, entering the era of artificial intelligence, scholars have gradually made intelligent sports a new technological science through the development and simulation of intelligent sports and the improvement and optimization of the theoretical system of intelligent sports.

### 2.3. Application of Intelligent Sports

The application of artificial intelligence in sports mainly includes competitive sports and national fitness. In terms of competitive sports, Trawinski [9] studied the prediction accuracy of sports events based on intelligent model testing. Verlic et al. [10] used artificial intelligence to analyze the training content and nutrition supply of athletes. Albu and Stanciu [11] tried to provide sports medicine and sports rehabilitation for athletes after injury by using the technical method of artificial intelligence. In the field of national fitness, research focuses are mainly on fitness feedback, nutritious diet, and intelligent equipment. Wang and Yang [12] carried out research on the assessment of sports injury based on neural network. Novatchkov and other scholars [13] analyzed the training plan and training feedback of artificial intelligence strength training in the fitness process. National fitness is an effective means to prevent cardiovascular diseases. Baashar et al. [14] studied the influence of artificial intelligence on cardiovascular diseases. Silva [15] designed an exercise diet evaluation software to make people more scientific about fitness. Cai et al. [16] developed a composite material of carbon nanotubes with extendability as a motion sensor. In addition, major sports manufacturers have invested a lot of manpower and material resources in the R&D of intelligent sports equipment. For example, sports brands such as Nike, Li Ning, and Adidas have teamed up with Apple, Huawei, Xiaomi, and other technology giants to create intelligent wearable devices, bringing intelligent sports into people's daily lives.

## 3. Status of Intelligent Sports Development in National Fitness

### 3.1. Development Dilemmas

#### 3.1.1. Data Security Risks

The application of intelligent sports in national fitness mainly refers to data acquisition and collection through big data and cloud computing. However, the use of AI to do data statistics and locate bodybuilders will inevitably cause data security risks. Intelligent sports data security risks are divided into two types: active risk and passive risk. Taking smart fitness centers as an example, smart gyms record members' physical data and workout tracks, and also store members' basic information and consumption levels. Any behavior or movements of members in the centers will be stored as data. The data collected present a risk of being resold by gyms to other data-demanding enterprises (pharmaceutical enterprises, health care enterprises, etc.) through the backstage big data platform, which will virtually cause serious troubles to customers' privacy. We describe this privacy disclosure as active risks. As for passive risks, given that intelligent sports technologies are not mature enough, the data are mostly processed in a centralized way. This data-processing approach is easy to be attacked by hackers, causing the occurrence of network security events. Due to the worry that they will be tracked by big data, people would choose to reject and resist intelligent sports in life, which makes it difficult to popularize and apply intelligent sports in the process of national fitness.

#### 3.1.2. Market Monopoly

With the continuous application of intelligent sports in national fitness, basic data of national fitness have become important assets for the development of intelligent sports enterprises. Nevertheless, most of the assets are held by enterprises with solid capital, technology, and talent reserves. Intelligent sports giants make full use of the data to develop more targeted and scientific products, making themselves even more powerful. This will gradually lead to polarization, during which small and medium-sized intelligent sports companies eventually go bankrupt while leading enterprises continue to monopolize the market. It will not only cause market disorder of national fitness industry but also abate people's enthusiasm for bodybuilding.

#### 3.1.3. Legal Supervision

In China, Sports Law plays a key role in the development of the sports industry and national fitness, but there are few laws and regulations in the field of intelligent sports. With the continuous progress of the intelligent sports market, the market environment is becoming more and more severe. Vicious competition, lack of market supervision system, and the unfulfillment of market supervision are largely seen and constantly spreading, resulting in the malignant development of intelligent sports. Given a huge profit temptation in the market of national fitness, illegal acts such as piracy of intelligent products, copying of data, and privacy infringement occur from time to time. When violated, enterprises and individuals without legal protection have no place to safeguard their rights, which seriously flounders the market order and the high-quality development of the national fitness industry.

#### 3.1.4. Product Updating and Iteration

The development of intelligent sports mostly relies on technical products, and the upgrading of products will bring consumers better services and renewed experience. For both national fitness firms and individuals, excessive speed of product updating and iteration will bring some losses, and the “substitution effect” is particularly pronounced. Product updating is bound to affect the experience of consumers, reduce the service life of products, and also exert a certain negative impact on the popularization of national fitness.

### 3.2. Development Advantages

#### 3.2.1. Policy Guarantee

Nowadays, China is in the critical period of the implementation of national fitness, and thus fostering the intelligent development of national fitness is the future development trend and driving force. As mentioned in the 14th Five-Year Plan for Sports Development and many other public documents, China should vigorously develop the digital sports industry, promote cross-border integration of intelligent digital industries and sports industries, and accelerate the transformation and upgrading of sports through informatization, digitalization, and intellectuality. China has issued a number of policies and plans on intelligent sports to encourage and guarantee the extension of national fitness to the digital field, which is conducive for the rapid development of intelligent sports in the context of national fitness.

#### 3.2.2. Market Demand

With continuous popularization and application of science and technology, the public consumption level has been increased and keep-fit has become a popular lifestyle. At the same time, public demand for intelligent fitness is ever-increasing, and the market demand is correspondingly expanding, which will directly impress the value embodiment of intelligent sports in national fitness. In order to realize people's yearning for a better life, it is high time to explore the innovative development mode of intelligent sports and provide high-quality service supply to people. This will also help intelligent sports develop into a new stage of supply-demand balance and industrial maturity.

#### 3.2.3. Industrial Upgrading

As the development of intelligent sports deepens, the traditional sports industry is being transformed into a high-tech one. New industrial parks and industrial bases have realized fully automated production, packaging, and transportation. The application of intellectual technologies can largely improve product quality while reducing labor and material costs, gradually transforming and upgrading traditional sports manufacturing to a smart one. Industrial upgrading is beneficial in various aspects. As for enterprises, it can greatly raise their development prospect and potential by improving their production efficiency. With regard to consumers, it helps provide more accurate and personalized products and services, and stimulate new demand for sports consumption. From an industrial perspective, it may boost the national fitness industry to high-end manufacturing industry.

### 3.3. Research Significance

#### 3.3.1. Promotion of Public Health and Sports Market

To build a system of intelligent sports in national fitness helps conform to the new trend of national fitness development, speed up the integration of artificial intelligence and national fitness, promote the application and practice of intelligent sports, raise the health awareness of people, and generate public enthusiasm to participate in fitness. At the same time, the system can optimize the national fitness market to a certain extent, stimulate the market vitality, motivate the market innovative impetus, and improve the market competitiveness.

#### 3.3.2. Formation of a Data-Driven and Open Industrial System

The construction of intelligent sports system in national fitness can cultivate a data-driven industrial system. A national fitness data platform system based on big data and cloud computing will improve interconnection, coordination, and feedback efficiency of governments, markets, and citizens. In addition, the national fitness data are going to be open and shared, which is instrumental for governments to master first-hand data and real-time implementation of national fitness, and timely optimize and adjust implementary measures.

#### 3.3.3. Orientation to Innovation and Scientific Policies

The integrated development of artificial intelligence and national fitness can give full play to the active guidance of the government in planning and investing in the national fitness strategy, and further improve the policy-making on finance and market of the digital fitness industry. Furthermore, the full use of advanced technologies is conducive to thoroughly implementing the innovation-driven development strategy in national fitness, accelerating the application of intelligent sports in national fitness, and generating new technologies, formats, and models for national fitness.

#### 3.3.4. Better Management and Coordination of Social Subjects

By setting up an implementary system, the social subjects involved in national fitness can be better managed and coordinated, their multilateral relationship clarified, and their current and future trend mastered. Finally, the orderly implementation of national fitness strategy will come true. Moreover, by setting up a guarantee system in each link, the institutional and political support can be strengthened, the supervision of the national fitness industry perfected, the interests of all social subjects protected, and the market stability ensured.

## 4. Construction of Intelligent Sports System in National Fitness

As previously discussed, the application of artificial intelligence technology to national fitness has an essential role to play. For one thing, it can further accelerate the implementation of this national strategy by building a new development model, forming new ideas and providing new technological support for national fitness. For another, through national fitness statistics, intelligent sports can guide the public to scientific fitness, monitor the physical health of sports people, and generate the public enthusiasm for keep-fit. This paper presents a logic framework of intelligent sports system in national fitness (see Figure 1), where the basic situation and changes of national fitness are grasped through big data platform, and the real-time trends of national fitness are obtained through information technologies such as Internet Plus, Internet of Things, cloud computing, VR, and AR. In addition, national fitness bodies such as community sports, rural sports, school physical education, sports integration, and mass sports events will be subject to fine management, summary, feedback, guidance, guarantee, and planning. Finally, a national fitness data platform and a scientific fitness system for sportsmen and sportswomen will be formed.

### 4.1. Development Principles

#### 4.1.1. Scientificity

Intelligent sports must follow scientific principles in the implementation of national fitness strategy, and provide precise and effective services for national fitness through big data, cloud computing, and other science and technology. Intelligent sports products should ensure their safety, reliability, and protection of privacy. At the same time, intelligent sports should follow the industry rules and legal norms in the field of sports and artificial intelligence, and participate in the national strategy of national fitness scientifically, safely, legally, and effectively.

#### 4.1.2. Effectiveness

Internet Plus, Internet of Things, 5G, and other information technologies are the basis for the development of intelligent sports. Compared with traditional sports, intelligent sports has more R&D investment and production costs, so the principle of effectiveness should be respected. For one thing, fitness data collection, processing, analysis, and storage are highly efficient, which embodies the superiority of intelligent sports. For another, faster and better response to the needs of sports-lovers and more effective and scientific fitness services will also reflect the value and significance of intelligent sports.

#### 4.1.3. Public Welfare

In the strategy of national fitness, intelligent sports application should adhere to the interests of people, strictly abide by the moral code and legal norms, and resolutely prevent the loss of public interest. More specifically, as for public interest, intelligent sports should provide targeted services for people, formulate scientific fitness programs, monitor physical health in real time, and improve the sports rehabilitation system. As for national interest, it should provide convenience for government work, accurately grasp the situation of national fitness in various regions, and offer data reference for formulating more reasonable and effective national fitness plans. Last but not least, from the perspective of enterprises, it is expected to provide new opportunities for the development of enterprises, innovate their development paths, and enhance the protection of their intangible assets.

#### 4.1.4. Collaboration

Since intelligent sports itself is the fusion of two different fields, the cooperation and communication between various disciplines are therefore essential. It is necessary to strengthen interdisciplinary exchanges and optimize the integrated development system for multi-disciplinary industries, universities, and research institutes. In addition, since national fitness involves a wide range of social subjects with discrepancies, it requires subjects from different regions, departments, and organizations to enhance cooperation and enlarge exchanges in order to achieve a win-win situation.

### 4.2. Basic Framework of National Fitness Intelligent Sports System

As highlighted earlier, the engagement of intelligent sports in national fitness requires precision, intelligence, and interconnection, to make the implementation of this national strategy more comprehensive and smart. Based on this, we construct a content framework of national fitness intelligent sports system (see Figure 2) that is mainly composed of four layers:

1. Base layer. This is the basis for the application of artificial intelligence in the process of national fitness. Artificial intelligence relies on data, algorithms, and hashrate. The data are collected and transmitted by biosensor, photosensor, sound sensor, and chemical sensor. In China, more than 500 million residents regularly take part in physical exercise. The national fitness intelligent sports system is going to establish multiple data subsystems in each province and city. The total system supports data management of projects as large as 10PB, as well as multi-file, distributed storage. The data scale of each subsystem is determined by the system scale, ranging from 1TB to 10PB. The algorithm is to store and calculate through simulation training chip, cloud inference chip, and terminal device chip. The hashrate includes hashrate environment, scale, and application. The national fitness intelligent sports system is mainly funded and constructed by the government. The hashrate is applied to various fields of national fitness, such as intelligent service system, data management system, operation system, etc. The scales of hashrate are divided according to the service areas of each subsystem. The hashrate scales of national and provincial systems should reach the level of intellectual hashrate, supporting 10TFlops or 1000TFlops parallel computing system, as well as multi-node, CPU, multi-processor, and other multi-level parallel computing. Scales of hashrate of each subsystem should be chosen according to scales of database.
2. Data layer. The data layer is the core of the content framework of the national fitness intelligent sports system. It mainly involves data of three comprehensive fitness subjects: government (industrial data, organization data, planning data), society (fitness sites, human resources, events), and the people (fitness data, sports consumption, fitness security).
3. Management layer. This layer mainly includes database management, operations management, security management and data maintenance. The date are shared and communicated by public and private clouds of the hybrid cloud data storage system.
4. Application layer. The application layer indicates the ultimate goal and social significance of national fitness intelligent sports system. Here, technologies including artificial intelligence, computer vision, biometric recognition, natural language processing, automatic control, image processing, clustering and collaborative filtering technology, and information retrieval are applied to the following systems of national fitness data monitoring, statistics, guidance, and guarantee. At present, these applications are achieved in intelligent fitness venues, intelligent sports equipment, VR games, and training.

From the content framework of national fitness intelligent sports system, we can see that intelligent sports is of great value and significance for the implementation of national fitness. It is because the engagement of intelligent sports is of great help to accelerate and broaden the implementation from multiple perspectives, fields, and levels; provide more convenient and scientific fitness guidance for people; and eventually meet the people's growing demand for bodybuilding and their yearning for a better life.

### 4.3. Function Design of National Fitness Intelligent Sports System

From the perspective of intelligent sports itself, its functions mainly lie in data, calculation, and intelligence. Primarily, through a colossal database and high-speed computing, intelligent sports can simplify the government departments' tracking of the current situation and provide various indicators and information for national fitness policy-making. In addition, by offering portable and convenient work-out activities, it is helpful in innovating the traditional way of national fitness popularization, accurately feeding people's needs for sports and fitness, and effectively arousing public enthusiasm for national fitness.

From the perspective of national fitness, intelligent sports is a shortcut in the implementation of this national strategy, due to the fact that it can make measures more efficient and scientific, and make it easier for the public to accept fitness policies and activate fitness motivation. Since national fitness is a nation-wide strategy, involving people from different geographical locations, living environments, and social backgrounds, this huge project requires the help and participation of intelligent sports to better unify and coordinate.

The main functions of the national fitness intelligent sports system (see Figure 3) mainly include four layers: ①Data statistics and accurate services are carried out for sports fitness people, sports consumption level, and sports facilities. ②Scientific fitness programs are offered to active people by developing personalized fitness programs and on-site AI guidance. ③Fitness feedback and service guarantee are provided to active people by supervising their fitness behaviors, recording their fitness tracks, and instructing scientific bodybuilding methods. ④Sports products can be intellectually upgraded and public awareness of fitness aroused with the help of technologies such as intelligent equipment upgrading, AI fitness perception interaction, and 3D visual scene simulation.

#### 4.3.1. Data Statistics and Lean Services Provide Data Support for National Fitness

Data statistics and service is an important work of intelligent sports in the implementation of national fitness. From the perspective of governments, they calculate the proportion of people who regularly participate in physical exercise, their exercise frequency, intensity and approaches, use of sports facilities and sites, as well as their levels of sports consumption, etc. In doing so, governments can more accurately grasp the overall situation of national fitness. From the perspective of active people, intelligent sports can analyze personal fitness data to better monitor their own health and master personal fitness effects in real time. At the same time, intelligent sports helps provide sports lovers with reasonable products and avoid excessive consumption. In addition, people can observe the use of sports venues through intelligent sports equipment, and then reserve sports sites more conveniently and effectively, which will also improve the utilization and reduce the congestion of sports venues.

#### 4.3.2. Demand Guidance and Scientific Plan Provide Intelligent Services for National Fitness

Since the service object of national fitness is mainly the people, the main purpose of intelligent sports application in national fitness is to meet the public fitness needs. Fitness guidance and scientific fitness program are the urgent needs of people. Therefore, it is essential to understand people's fitness purpose, hobbies, leisure time activities, and so on through the intelligent sports big data platform, given that it can provide targeted scientific fitness programs, guide the public to participate in sports, avoid wrong movements and mistaken ways, and prevent people from sports injuries or other unnecessary dangers. The superiority of intelligent sports lies in one-to-one service. Thanks to VR, 3D, and other virtual technologies, people can experience simulated training in a multi-scenario and multi-perspective way, which changes the traditional, generalized, and random way of workout. For example, the elderly with heart disease, osteoporosis, and hypertension are not suitable for medium and high-intensity training.

#### 4.3.3. Fitness Feedback and Service Guarantee Provide Intelligent Protection for National Fitness

At present, a serious shortage of social sports instructors in China leads to difficulties of pre-fitness guidance, post-fitness feedback, and rehabilitation of sports injuries. In the face of the current situation, monitoring fitness behavior and recording fitness track by intelligent sports can solve these problems. In addition, the establishment of fitness feedback and protection system with artificial intelligence can largely help fitness people know more about sports, master more exercise skills, and well control their fitness situation. The service of sports rehabilitation provided by intelligent sports may give less sense of reality for costumers, but the service area is large, the audience is of wide range, the input of manpower and material resources is reduced, and the controllability of the service is enhanced.

#### 4.3.4. Product Upgrading and Interest Stimulation Provide Innovative Power for National Fitness

By constantly upgrading fitness products, intelligent sports can optimize product performance and services, make sports equipment more intelligent and smart, and provide innovative technologies and means for national fitness. Along with the ongoing public adaptation to high-tech intelligent fitness products, people will gradually take physical exercise as an essential part of life. That is how intelligent sports stimulates public enthusiasm and generates public motivation for national fitness. In addition, the function of interactive communication is very easy for people to try, which is conducive for enhancing their affection between friends and relatives, and forming a sustainable and regular way of fitness. The 3D visual simulation technology adopted by intelligent sports can infect and mobilize people around to try workout and finally form the habit of fitness.

### 4.4. Content Design of Intelligent Sports System for National Fitness

The core of intelligent sports application in national fitness is to build an intelligent data platform for national fitness (see Figure 4). The platform is mainly composed of three subjects: (1) sports government departments. The sports government department is the executor and guide of the national strategy of national fitness. With the help of the intelligent sports system, fitness centers in various regions can facilitate venue reservation, physical monitoring, and equipment management, so as to ensure the basic fitness needs of the public. At the same time, these fitness centers can make statistics on sports venues, people's interest and fitness situation, and then summarize them to the corresponding sports departments. Therefore, the sports department levels can grasp the basic situation of the national fitness in their regions, timely adjust and improve the national fitness plan, and ensure the completion of comprehensive fitness with high quality through the statistics of various sports industry data and administrative data. (2) Sports social organization. Sports social organizations serve as a link in the strategy of national fitness. Sports associations are expected to use the intelligent sports system to organize and promote various sports events and public sports activities, and motivate people to participate in sports. Meanwhile, private, nongovernmental sports units with AI technologies can practice technical innovation, innovative production, and achieve industrial transformation and upgrading, so that their speed of development, potential, and competitiveness will be boosted. Also, sports foundations are expected to use intelligent sports systems to manage and calculate their finances, which will greatly improve the efficiency of foundations and help them better serve the society. (3) Fitness people. Fitness people are the foundation of national fitness strategy and the main object of intelligent sports service. People who workout regularly are divided into three groups: middle-aged and elderly fitness group (≥45 years old), youth fitness group (18–44 years old), and children fitness group (≤17 years old). Different age groups should adopt different fitness programs, carry out different fitness guidance, take different health monitoring means, participate in different fitness activities, develop different sports rehabilitation plans, etc. The collection of fitness data of different age groups can help governments to formulate more reasonable national fitness plans and install more useful fitness facilities. Meanwhile, it can help social sports organizations to hold different events, manufacture different products, and adopt more favorable fund support measures according to fitness conditions of different age groups.

### 4.5. Operation Analysis of National Fitness Intelligent Sports System

Intelligent sports is a very complex system in the implementation of national fitness strategy, which involves a large number of people and a wide range of fields. It is necessary to divide intelligent sports into different subsystems. The intricate cooperation, communication, and transformation relationship between each subsystem forms the intelligent sports system and a clear operation mechanism of national fitness. The operation mechanism of the national fitness intelligent sports system (see Figure 5) mainly includes the operation among social subjects of national fitness and the data operation system of national fitness.

#### 4.5.1. Operation Mechanism of Social Subject

The government department is taken as a pivot for the operation mechanism of social subject of national fitness intelligent sports. Sports government departments need to establish a system for integrated cooperation to better coordinate and cooperate with other social subjects and optimize government management. There is a two-way operation mechanism between governments and other social subjects, which means integrating government departments to formulate national fitness plans and policies for sports enterprises, associations, and the public. Meanwhile, enterprises, communities, social organizations, and the public provide feedback and suggestions on policy planning. At the same time, the government establishes a national fitness talent pool system to provide research projects for talents and expert teams. Conversely, this system also provides expert advice and evaluation for comprehensive fitness planning and policy-making. The operation mechanism of social subject is the basis and guarantee of the intelligent sports system of national fitness, which can motivate all social subjects of national fitness and facilitate the construction of the basic operation system of national fitness.

#### 4.5.2. Data Operation Mechanism

Data operation is the center of intelligent sports in the implementation of national fitness. It mainly includes: ①Data input. Firstly, the social subject mechanism provides data of national fitness. Secondly, the intelligent sports big data platform collects all basic data, and then carries out data mining and data feedback for different levels of departments. Finally, the intelligent sports big data platform inputs them into the national fitness big data platform. ②Data statistics and analysis. Relevant data input from the national fitness data platform will be fed back to government departments for data reference, which will help departments to summarize current implementation of national fitness. Then, departments will optimize and analyze the data, and finally build a data application model. ③Data output. Through data input and analysis, the data will finally be put into practice and application. After that, the superior departments will be fed back and suggested. Lastly, government departments will evaluate the optimized data and adjust and improve the existing national fitness plan.

#### 4.5.3. Intermediary Mechanism

The intermediary mechanism of national fitness intelligent sports system is the internal connection center between the operation data and social subjects, and also the link of the whole system. Firstly, the operation system of social subject collects and summarizes the basic data collected from citizens, markets, and industries through the intermediary mechanism, and transmits them to the database to realize data supply; The database classifies and processes all kinds of data to social subjects through the intermediary mechanism to meet the data needs. Second, the intermediary mechanism preprocesses the data through data stratification, makes statistics and analysis of the processed data, and stratifies and analyzes the national fitness data according to social groups and application fields, so as to improve the processing efficiency of the database. Thirdly, the intermediary mechanism analyzes and manages the whole operation mechanism, reduces operation errors and data processing errors, protects data privacy, and ensures data security. Fourthly, the intermediary mechanism optimizes information processing and information induction, carries out information integration for the overall operation mechanism, and then outputs the final data according to the application objectives. The relationship between data demanders is sorted out in an orderly manner, which greatly improves the cooperation between operating units and achieves information sharing.

## 5. Analysis on the Application of National Fitness Intelligent Sports System Taking Intelligent Fitness Center as an Example

### 5.1. Content Analysis of Intelligent Fitness Center

#### 5.1.1. Infrastructure

The basic facilities of the intelligent fitness center are more intelligent and scientific, which can better meet the needs of active people for fitness, improve the quality of fitness service and fitness experience. Firstly, the Internet of Things will be used to intelligently monitor and manage the service efficiency, site maintenance, automatic temperature control and humidity control, and light adjustment of the venue's placement information sensors, temperature sensors, and photosensitive sensors. Secondly, the intelligent fitness center uses the chip to install a series of auxiliary training equipment for sports, which can help green hands master the correct movement and improve fitness efficiency. In addition, smart fitness center provides more convenience and better service for fitness people through APP, SaaS, and IoT intelligent hardware. Finally, the intelligent fitness center has the management and control platform of the whole venue, which is responsible for the operation and maintenance of the whole venue, and can grasp the dynamic of the venue in real time to understand the fitness needs. It can also provide a series of service platforms such as venue reservation, face recognition, and fitness monitoring and tracking.

#### 5.1.2. Data Collection and Processing

The infrastructure collects data through sensors, chips, and data platforms and feeds it back to the data layer. Smart fitness center collects data of fitness people, venues, and sports events through artificial intelligence, Internet of Things, big data, and other science and technology. Data collected mainly include fitness intensity, sports consumption level, venue utilization, venue management, and so on. The data system processes and classifies the collected data, and finally feeds back the collected data to the management layer.

#### 5.1.3. Venue Management

Various data regarding venues collected by intelligent fitness center through the data layer are going to be applied to the venue management system. First, the intelligent fitness center database conducts data storage, retrieval, application, and transformation, and establishes an intelligent fitness center database system. Secondly, the data feedback from the data layer is used to find the loopholes and deficiencies in venue management, operation, and facilities, timely adjusting the management system and maintaining facilities. Finally, the establishment of data security maintenance system is to prevent data leakage or infringement on the privacy of fitness people, and protect the rights and interests of intelligent fitness center.

#### 5.1.4. Venue Application

Through the management of data and technology, data, technology, and management mode are put into practice. The first step is to establish the fitness monitoring and tracking system of members according to the national fitness data. The second step is to develop one-to-one fitness guidance programs based on the AI intelligent system, and provide fitness suggestions and exercise prescriptions specifically to meet the fitness needs of members. The third one is to use new technologies to create VR panoramic experience, simulated training, and fitness interaction to enhance the enjoyment of fitness and arouse fitness enthusiasm. Fourthly, to develop a set of management system suitable for the fitness center itself, which is based on the venue management data feedback. This is of help for reducing the operating cost and improving the intelligent level of the venue.

### 5.2. Function Design of Intelligent Fitness Center

#### 5.2.1. Data Statistics and Analysis

Intelligent fitness center operation and management are inseparable from data statistics and analysis, in that customer service, venue operation, facility usage, and flow monitoring all need data support. In addition, the consumption data of intelligent fitness center can help understand bodybuilders' consumption level, provide diversified services, and adjust service content in time. In addition, the smart fitness center summarizes its data to the fitness data platform of the local government, providing data support and reference for the formulation of national fitness plan.

#### 5.2.2. Scientific Guidance and Services

The essential function of intelligent fitness center is to provide fitness services for fitness people. First, in accordance with the needs, goals, and physical conditions of different fitness groups, intelligent fitness center develops targeted fitness programs and exercise prescriptions. Second, intelligent fitness center provides AI guidance or professional coach for fitness instruction to prevent sports injuries and ensure a scientific and effective way of fitness. Third, intelligent fitness center provides guidance for venue services, including venue reservation, event information, venue navigation, which can be achieved by APP, Wechat official account, and SaaS.

#### 5.2.3. Health Assurance and Feedback

The intelligent fitness center should ensure the health of the fitness people, and timely optimize and improve the potential safety hazards. When there are sports injuries or safety problems in the fitness center, professional trainers, with the help of intelligent equipment, judge the state of injuries, formulate corresponding physical treatment, and keep tracking the injured through AI. In addition, the intelligent fitness center summarizes and uploads the data to data platforms at higher levels. The superior platform also feeds back the data after processing to the intelligent fitness center data platform for improving services and adjusting optimization plans.

### 5.3. Operation Mechanism of Intelligent Fitness Center

#### 5.3.1. Operation Analysis of Different Subjects of Intelligent Fitness Center

Intelligent fitness center has a multi-tiered relationship with social subjects, including bodybuilders, venue operators, sports associations, and sports government departments. Fitness people are its main service object. Venue operators are responsible for the management, operation, and maintenance of the venue. Sports associations organize all kinds of mass sports events and sports activities in the fitness center. Government departments conduct overall planning and top-level designs for intelligent fitness center. As we can see, the four subjects are interconnected. According to the service to fitness lovers and sports associations, venue operators collect relevant data and feedback, and constantly optimize venue infrastructure and intelligent services; At the same time, venue operators feed back the information to government departments, which process and summarize the information through the talent pool system, adjust and optimize the national fitness plan, and feed back again to the intelligent fitness center.

#### 5.3.2. Operation Analysis of Intermediary Mechanism of Intelligent Fitness Center

The intermediary mechanism of intelligent fitness center is jointly constructed by data platform and venue operators. The data platform of intelligent fitness center stores and classifies the basic fitness data, preprocesses simply the data, and then transmits them to a higher level government database system. Finally, different data processing is carried out according to different application purposes. Venue operators are intermediaries connecting all social subjects, meeting the needs of fitness people, providing precise services, and operating the fitness center under the management and coordination of the government. The data information platform and operators jointly build an intermediary mechanism which meets the operational and managerial needs of the entire intelligent fitness center system and becomes the connection center and link of the system.

#### 5.3.3. Data Operation Analysis of Intelligent Fitness Center

Data operation of intelligent fitness center represents the core of the whole system. First of all, the data of fitness people and venue are collected through Internet of Things, AI, Internet, and other technical means, and uniformly summarized to the data platform of fitness center. Then, the fitness center platform is used to process the data. Part of the data statistics of the venue is used by itself for venue optimization, and others are uploaded to the superior government database for further application and practice. Finally, the superior database processes the data, conducts in-depth analysis according to the application purpose and direction, and then constructs a corresponding model which will be applied into the national fitness plan, realizing the transformation and utilization of national fitness achievements.

## 6. Development Strategy of Intelligent Sports in the Implementation of National Fitness

### 6.1. Optimize the Top-Level Design of Intelligent Sports Government

The top-level design and theoretical and practical system construction for the development of intelligent sports should be a high priority. First, formulate more perfect and specific development plans for national fitness intelligent sports to guide the future development direction and objectives of intelligent sports. Second, fill the gaps in laws and regulations related to intelligent sports, establish a scientific legal system, so that there are laws to follow, and the development rights and interests of intelligent sports in national fitness can be protected. Third, government departments should increase their support for intelligent sports enterprises by establishing funds to encourage the development of small, medium-sized, and micro enterprises. Meanwhile, they are supposed to establish a cooperation mechanism between large enterprises and small, medium-sized, and micro enterprises for their mutual benefit, and give play to the leading and exemplary role of sports giants.

### 6.2. Accelerate the Transformation and Upgrading of Intelligent Sports Industry

The transformation and upgrading of intelligent sports industry are key to the implementation of national fitness strategy. First, give full play to the distinctive characteristics of the intelligent sports industry as specialization, precision, speciality, and innovation to improve the core competitiveness of the sports industry. Second, build a development model of industrial chain and enhance the controllability of the industrial chain and form a vertical ecosystem of the industrial chain. Focus on key industrial domains such as sporting goods manufacturing industry, fitness industry, tourism service industry, and information industry. Accelerate the construction of intelligent sports integration system, which includes multi-industrial combinations of intelligent sports with medical industry, tourism, and health industry. Third, construct a standard system of the intelligent sports industry, create a comprehensive pilot work of national standards, promote the industrial quality standards of intelligent sports equipment and high-end equipment, and establish a collaborative mechanism of intelligent sports standards. Fourth, facilitate the innovative application of emerging technologies such as cloud computing, big data, Internet of Things, Internet, VR, and 5G in intelligent sports, and encourage the public sharing of data owned by intelligent sports enterprises. Build a multi-level and multi-link application system, improve the level of industrial intelligence, construct a digital transformation and upgrading mechanism, and enhance the supply capacity of intelligent sports transformation services.

### 6.3. Construct an Intelligent Sports Market Supervision Mechanism

The bottleneck of intelligent sports development needs to be assisted by market operation and supervision. There are great loopholes in the supervision of intelligent sports market, which leads to illegal vendors making huge profits through various means, resulting in the chaos of the market environment. First, the intelligent sports technology should reinforce the privacy security and protection for public interests to avoid potential security risks caused by its own vulnerabilities. Second, government departments and social subjects have to jointly build an intelligent sports security protection system, punish more severely unlawful acts such as infringement and market monopoly, and establish a market oversight committee to regularly inspect and supervise the intelligent sports market. Third, strengthen safety publicity, raise people's awareness of intelligent sports products, strengthen people's legal awareness of intelligent sports, and achieve “universal supervision and common resistance.”

### 6.4. Establish an Intelligent Sports Talent Training System

Given that talents are fundamental for the development of intelligent sports, establishing a good talent training system is an important step for the sustainable development of intelligent sports. First, tap high-end talents of intelligent sports. At present, China is seriously lacking integrated talents of “artificial intelligence + sports.” Experts and scholars in relevant fields at home and abroad should be attracted to enter the intelligent sports industry to provide advanced technical experience. Second, promote the coordinated development of governments, industries, and universities, and that of research and application. Take the intelligent sports market as the leading factor and use government policies to drive the cultivation of intelligent sports talents. Then, establish an intelligent sports innovation platform, introduce high-quality intelligent sports enterprises, encourage efficient and scientific research institutions to strengthen intelligent sports research, and promote the transformation and practical application of innovative achievements to release the vitality of the industry. Third, establish an intelligent sports talent training mechanism. Establish a joint training and development system through four different social subjects: government, market, enterprises, and universities. Rely on the sports science and technology innovation platform, strengthen cooperation and exchange, and create a talent training mode of sustainable output to ensure the positive role of intelligent sports in national fitness.

## 7. Conclusion

In recent years, the national strategy of national fitness in China has made breakthroughs, and intelligent sports in national fitness has been applied widely, showing great potential and motivation. Intelligent sports applications such as VR games have become one of the important ways for the public to participate in national fitness. With the support and encouragement of various Chinese policies, intelligent sports will surely become the core of the development of the strategy for China to become a sport power in the future. In the development of intelligent sports and national fitness, it is necessary to analyze the opportunities and risks generated by intelligent sports in a dialectic way. We need not only to recognize the superiority and advancement of intelligent sports but also to fully understand the challenges of intelligent sports on the market economy and society. This research indicates that building the national fitness intelligent sports system is the foundation of intelligent sports engagement in national fitness implementation. This study analyzes the logic, framework, content, and operation of intelligent sports system in the national fitness theoretically and practically. It also demonstrates that intelligent sports gives full play to the value of advanced technologies such as big data, Internet in fitness business. The implications of this article are the following. Social subjects should analyze the application of intelligent sports from multiple perspectives, minimize the risks brought about by intelligent sports when enjoying the convenience and effectiveness. Also, the market system ought to be improved, the top-level design enhanced, comprehensive talents of “intelligence + sports” cultivated, in order to speed up the great goal of making China a sports power.

## Figures and Tables

**Figure 1:** Logic framework of intelligent sports system in national fitness.

**Figure 2:** Content framework of national fitness intelligent sports system.

**Figure 3:** Main function design of national fitness intelligent sports system.

**Figure 4:** Content structure of national fitness intelligent sports system.

**Figure 5:** Operation mechanism of national fitness intelligent sports system.

## Data Availability

The dataset used in this paper is available from the corresponding author upon request.
